This article has been retracted.

# Examining the effects of information and communications technology on green growth and environmental performance, socio-economic and environmental cost of technology generation: A pathway toward environment sustainability

**DOI:** 10.3389/fpsyg.2022.999045

**Published:** 2022-09-12

**Authors:** Shaoming Chen, Muhammad Tayyab Sohail, Minghui Yang

**Affiliations:** ^1^International Business School, Guangzhou City University of Technology, Guangzhou, China; ^2^School of Economics and Trade, Guangdong University of Foreign Studies, Guangzhou, China; ^3^School of Public Administration, Xiangtan University, Xiangtan, Hunan, China; ^4^South Asia Research Centre, School of Public Administration, Xiangtan University, Xiangtan, Hunan, China; ^5^Research Center for Accounting and Economic Development of Guangdong-Hong Kong-Macao Greater Bay Area, Guangdong University of Foreign Studies, Guangzhou, China

**Keywords:** ICT penetration, human capital, green growth, environment, technology generation

## Abstract

Human capital and ICT have a significant role in determining human development. The impacts of ICT and human capital on green growth and environmental sustainability should be explored for sustainable economic development. This research contributes to the literature on the role of ICTs and human capital in the determination of green growth and environmental performance. Based on time-series data 1990–2019, the study intends to investigate the impact of ICTs and human capital on environmental and green growth performance for China. The study reports that ICTs tend to reduce CO_2_ emissions and improve green growth in the long-run. However, education reduces CO_2_ emissions in the long-run but does not produce any significant impact on green growth in the long-run. It is suggested that government should invest in environmental efficiency and environmental technologies simultaneously with human capital that could significantly contribute to pollution reduction. Lastly, policies to increase human capital should be implemented simultaneously with policies to promote ICTs contribution in order to confirm green growth and environmental protection.

## Introduction

Over the past few decades, the world community has been striving to achieve the targets of sustainable development and the protection of the environment. However, the main hurdle in the way of the said targets is the extraordinary rise in the emissions of greenhouse gasses due to the enormous increase in consumption and production activities since the industrial revolution. Therefore, human activities are to be widely recognized as a major culprit in deteriorating the environment and disturbing the balance of the ecosystem (Kamonja et al., 2014; Usman et al., 2020; Sohail et al., 2021b,c, 2022c; Lan et al., 2022; Li et al., 2022a,b). Now the world has realized the existence of the problem of global warming and climate change, and the focus has been shifted to estimate the effects of such changes on the environment and the factors that can mitigate such effects and may have impacts on our environment (Yen et al., 2017, 2021; Yat et al., 2018; Yasara et al., 2019; Zhao et al., 2019, 2022a,b; Zhenyu and Sohail, 2022). Human activities are continuously damaging the environment, and if the process of environmental degradation continues, the existence of mankind on the planet earth will be jeopardized. To counter such damages the international community first signed Kyoto Protocol in 1998 and then Paris pact in 2015, both these agreements call for environmental protection by making activities of economic growth pro-environment and carbon-free. In this regard, Goal 13 of the sustainable development by the United Nations also emphasized quick and prompt actions to reduce CO_2_ emissions and to protect the environment (Undp, 2019).

In recent years, the concept of green development has emerged, which refers to uncoupling economic growth from CO_2_ emissions. Attaining cleaner production and green supply chain by controlling the production and consumption-driven emissions by employing green technological innovations also fall in the purview of green development (Porter and Van der Linde, 1995; Carolan, 2004; Ullah et al., 2021). Green growth also helps save energy and reduce carbon emissions (Sohail et al., 2013, 2019b,2021a; Guo et al., 2018; Arif and Sohail, 2020; Chai et al., 2021; Jian et al., 2021; Jiang et al., 2021) and is widely considered an important strategy to mitigate the severe impact of climate change. Green growth is crucial to attain production efficiency and decouple the economic growth from CO_2_ emissions, and during this process, green growth relies on factors such as technological and market innovations. Green technology can serve as a driver of green economic development (Sohail et al., 2020, 2021d,2022b,2022d; Sun et al., 2020), and the deployment of green technologies can curb the flow of carbon emissions (Usman et al., 2021). In this regard, the term “IT for green” can help to explain the grayish dimension of information technology (IT) (Faucheux and Nicolaï, 2011). This term describes how the IT sector can successfully curb CO_2_ emissions by integrating energy-efficient resources in different sectors of the economy (Usman et al., 2021).

ICT has played an essential role in the complete transformation of human society. Its role in the development of developing and emerging nations cannot be ignored (Salahuddin and Alam, 2016). Over the past few decades, the spread of the internet has completely overhauled the lifestyle of people by converting it into a digital one. The internet revolution has changed the perspective of looking at different things such as books, compact and check books converted into bytes, MP3s, and clicks. Further, efficient use of online shopping, e-commencing, teleconferences, and teleworking have made it possible to save time, money, and resources (Sui and Rejeski, 2002; Mustafa et al., 2021, 2022d,e). The migration of the economy from carnal to information capitals helps improve environmental feature and reduce energy consumption, a sign of a weightless economy that demands less capital for operation (Ozcan and Apergis, 2018; Huang et al., 2022; Khan et al., 2022, 2021; Zahid et al., 2022a,b). The said transformation has reduced the reliance of economies on physical resources for their growth process, reducing pollution emissions. For instance, online shopping, virtual classrooms, teleconferencing, and teleworking are all helpful in decreasing the use of transportation and travel services and gatherings at the shopping malls, which causes the energy consumption and CO_2_ to fall and may have impacts on resources (Muhammad et al., 2014; Shahab et al., 2016; Mahfooz et al., 2017, 2019, 2020; Rasool et al., 2017; Mustafa et al., 2022f).

Although there is consensus among the empirics regarding the positive relationship between ICT and economic growth; however, the relationship between ICT and CO_2_ emissions is debatable. Over the last three decades, the consumption and usage of ICTs have been on the rise, which is surging the energy demand. As a result, since the last few decades, the global energy demand has maintained a growth rate of 7% per annum (Salahuddin and Alam, 2016). Therefore, till the year 2012, the share of ICT in global CO_2_ emissions has reached 2% (The Greenpeace International, 2014). On one side, the large-scale production of ICT material contaminates the environment by emitting CO_2_ emissions (Wen et al., 2021). Similarly, the consumption of ICT products such as internet devices, cell phones, computers, laptops, smart TVs, etc., has augmented the energy demand (Moyer and Hughes, 2012). Thus, ICT-related emissions are coming from the production as well as demand side, which is the primary reason for the negative effects of ICT on CO_2_ emissions (Salahuddin and Alam, 2016).

Apart from ICT, human capital also transforms the economy’s production function by making it more human-capital intensive which will consume less energy than physical-capital intensive techniques of production (Sohail and Delin, 2013; Sohail et al., 2014a,b, 2015, 2019a,2022a; Jian et al., 2021; Li and Ullah, 2021). Human capital can influence the environmental quality and sustainable development. For instance, Chankrajang and Muttarak (2017) observed that human capital plays an essential role in the alteration of people’s attitudes that induces them to use renewable energy sources. Besides, the contribution of education in comprehending the causes and consequences of climate change cannot be undermined (Yin et al., 2021; Liu N. et al., 2022; Liu Y. et al., 2022; Lu and Sohail, 2022; Mustafa et al., 2022a,b,c). According to Sarkodie et al. (2020), education positively affects recycling activities. Bano et al. (2018) pointed out that human capital is crucial for promoting energy efficiency by modifying people’s behavior and creating awareness, which in turn reduces CO_2_ emissions. In the light of the above discussion, we have tried to analyse the impact of ICT and human capital on green growth and CO_2_ emissions for China.

## Model and methods

Ecological modernization theory noted that ICTs are considered a key factor of economic growth that leads to positive structural change that can reduce CO_2_ emissions (Buttel, 2000; York et al., 2010). The role of human capital is vital in determining green growth. ICT and education have positive economic externalities as well. Indeed, ICT and human capital are important factors in the green production processes by mitigating CO_2_ emissions. Following earlier theoretical and empirical literature Jacobs (2012), Sinn (2012), Song et al. (2019), Lahouel et al. (2021), and Usman et al. (2021), noted that the main determinants of green growth and CO_2_ emissions are ICT, education, renewable energy consumption, trade and financial development, Therefore, we initiate with the following models:


(1) $${\text{GG}}_{\text{t}}=\mu_{0}+\mu_{1}\,{\text{ICT}}_{\text{t}}+\mu_{2}\,{\text{Education}}_{\text{t}}+\mu_{3}\,{\text{REC}}_{\text{t}}+\mu_{4}\,{\text{FD}}_{\text{t}}+\mu_{5}\,{\text{Trade}}_{\text{t}}+\varepsilon_{\text{t}}$$

(2) $${\text{CO}}_{2,t}=\mu_{0}+\mu_{1}\,{\text{ICT}}_{\text{t}}+\mu_{2}\,{\text{Education}}_{\text{t}}+\mu_{3}\,{\text{REC}}_{\text{t}}+\mu_{4}\,{\text{FD}}_{\text{t}}+\mu_{5}\,{\text{Trade}}_{\text{t}}+\varepsilon_{\text{t}}$$

Equations 1, 2 are green growth (GG) and CO_2_ emissions (CO_2_) that depend on information and communications technology (ICT), educational attainment (Education), renewable energy consumption (REC), financial development (FD), and trade openness (Trade). The rise in ICT improves green development by reducing CO_2_ emissions, thus, an estimate of μ_1_could be positive (negative) in green growth (CO_2_ emissions) models. Education also has positive effects on green growth in reducing CO_2_ emissions. The expected estimate of μ_2_ to be positive in green growth and negative in CO_2_ emissions models. Estimates of μ_1_,μ_2_,μ_3_,μ_4_,*and*μ_5_ refect long-run effects of exogenous variables on green growth and CO_2_ emissions. Equations 1, 2 are provides long-run effects, but they cannot report short-run effects. An econometric approach that yields the long-run and the short-run effects in one step is that of Pesaran et al. (2001) as follows:


(3) $$\Delta \,{\text{GG}}_{\text{t}}=\mu_{0}+\sum_{\text{k}=1}^{\text{n}}\beta_{1\,k}\,\Delta \,{\text{GG}}_{t-k}+\sum_{\text{k}=0}^{\text{n}}\beta_{2\,k}\,\Delta \,{\text{ICT}}_{t-k}+\sum_{\text{k}=1}^{\text{n}}$$

$$\beta_{3\,k}\,\Delta \,{\text{Education}}_{t-k}+\sum_{\text{k}=0}^{\text{n}}\beta_{4\,k}\,\Delta \,{\text{REC}}_{t-k}+\sum_{\text{k}=1}^{\text{n}}\beta_{5\,k}\,\Delta \,{\text{FD}}_{t-k}+$$

$$\sum_{\text{k}=1}^{\text{n}}\beta_{6\,k}\,\Delta \,{\text{Trade}}_{t-k}+\mu_{1}\,{\text{GG}}_{t-1}+\mu_{2}\,{\text{ICT}}_{t-1}+\mu_{3}\,{\text{Education}}_{t-1}$$

$$+\mu_{4}\,{\text{REC}}_{t-1}+\mu_{5}\,{\text{FD}}_{t-1}+\mu_{6}\,{\text{Trade}}_{t-1}+\lambda .{\text{ECM}}_{t-1}+\varepsilon_{\text{t}}$$

(4) Δ⁢CO2,t=μ0+∑k=1nβ1⁢k⁢Δ⁢CO 2,t-k+∑k=0nβ2⁢k⁢Δ⁢ICTt-k+∑k=1n

$$\beta_{3\,k}\,\Delta \,{\text{Education}}_{t-k}+\sum_{\text{k}=0}^{\text{n}}\beta_{4\,k}\,\Delta \,{\text{REC}}_{t-k}+\sum_{\text{k}=1}^{\text{n}}\beta_{5\,k}\,\Delta \,{\text{FD}}_{t-k}+$$

$$\sum_{\text{k}=1}^{\text{n}}\beta_{6\,k}\,\Delta \,{\text{Trade}}_{t-k}+\mu_{1}\,{\text{CO}}_{2,t-1}+\mu_{2}\,{\text{ICT}}_{t-1}+\mu_{3}\,{\text{Education}}_{t-1}$$

$$+\mu_{4}\,{\text{REC}}_{t-1}+\mu_{5}\,{\text{FD}}_{t-1}+\mu_{6}\,{\text{Trade}}_{t-1}+\lambda .{\text{ECM}}_{t-1}+\varepsilon_{\text{t}}$$

where coefficient estimates β_1k_, β_2k_, β_3k_, β_4k_, β_5k_,and β_6k_reveal short-run impacts and estimates of μ_1_,μ_2_,μ_3_,μ_4_,μ_5_, and μ_6_are long-run impacts. An earlier study by Undp (2019) recommends two tests to establish cointegration, such as diagnostic tests (e.g., F-test and ECM). Previous conventional methods require that the variables of the model must be either stationary at I(0) or, at I(1). However, the ARDL model considers the mixture of I(1) and I(0) variables. Another privilege of the ARDL model is that it simultaneously provides long-run and short-run estimates. Additionally, a smaller number of observations is a common problem of time-series analysis. The advantage of the ARDL model is that it deals with the issue of a small number of observations and provides unbiased and efficient results. For unit root testing purposes, we have to employ Dickey Fuller-Generalized Least Square (DF-GLS). In the last stage, we also employ some diagnostic and stability tests. To check the problems of serial correlation, functional misspecification, Heteroskedasticity, we have applied LM, Ramsy’s RESET, and BP tests. The renowned CUSUM and CUSUM-sq tests are also applied to confirm short-term and long-run coefficient estimates stability.

## Data

This research examines the role of ICT and human capital on green growth and environmental performance for China over the period 1990–2019. Detail about definitions and symbols of variables and sources of data are given in Table 1. Green growth in this study is measured by environmentally adjusted multifactor productivity, while environmental performance is measured by CO_2_ emissions in kilotons. ICT index is measured by using internet users (% of population), mobile cellular subscriptions (per 100 people), and fixed telephone subscriptions (per 100 people). Human capital is measured by education in terms of average years of schooling. Besides ICT and education, the study has used some important control variables such as renewable energy consumption, financial development index, and trade as a percent of GDP. Data for green growth is scrutinized by OECD. The source of data for CO_2_ emissions and trade is the World Bank. The source of data for education is Barro and Lee, EIA is for renewable energy consumption, but ICT index data is calculated by the authors.

**TABLE 1:** Variable description and sources.

Variable	Mean	SD	Definitions	Sources
Green growth	9.297	1.688	Environmentally adjusted multifactor productivity	OECD
CO_2_	15.49	0.547	CO_2_ emissions (kt)	World Bank
ICT	27.23	25.03	ICT index	Authors calculation
Education	11.25	2.137	Average years of schooling	Barro and Lee
REC	6.501	5.569	Total energy consumption from nuclear, renewables, and other (quad Btu)	EIA
FD	0.459	0.114	Financial Development Index	IMF
Trade	43.06	10.54	Trade (% of GDP)	World Bank

## Results and discussion

Before executing regression analysis, the study tested the unit root properties of data. Thus, the dickey-fuller generalized least square (DF-GLS) test and augmented dickey-fuller (ADF) with structural break test have been used. The findings of both unit root tests have been displayed in Table 2. According to the DF-GLS test, green growth and ICTs are I(0) stationary, whereas CO_2_, education, renewable energy consumption, trade, and financial development are I(1) stationary. According to ADF with the unit root break test, green growth, CO_2_, ICTs, renewable energy consumption, and trade are I(0) stationary, whereas education and financial development are I(1) stationary. A mixture of I(0) and I(1) order of integration allows us to employ the ARDL approach for estimating the long-run cointegration relationship.

**TABLE 2:** Unit root test.

	I(0)	I(1)	Decision	I(0)	Break date	I(1)	Break date	Decision
Green growth	−2.756***		**I (0)**	−4.412*	2007			**I (0)**
CO_2_	0.752	−2.586**	**I (1)**	−4.965***	2002			**I (0)**
ICTS	−1.725*		**I (0)**	−10.25***	1994			**I (0)**
EDUCATION	0.275	−4.412***	**I (1)**	−2.102	2003	−4.563**	2017	**I (1)**
REC	0.102	−3.774***	**I (1)**	−5.576***	2014			**I (0)**
FD	0.245	−4.361***	**I (1)**	−2.256	2001	−5.745***	2001	**I (1)**
TRADE	−1.212	−3.485***	**I (1)**	−4.412*	2007			**I (0)**

***p < 0.01, **p < 0.05, *p < 0.1, respectively.

Table 3 reported ARDL estimates of CO_2_ emissions and green growth models. The long-run results of the green growth model report that ICT displays a positive effect on green growth while education reports an insignificant impact on green growth. It reveals that ICT contributes significantly to the determination of green growth, thus ICT development is embraced green growth. The coefficient estimate of the ICT displays that a 1 percent increase in ICT increases green growth by 1.284 percent in China. Our findings reveal that ICT tends to increase green growth. Nguyen et al. (2019) support our findings by arguing that the increase in the utilization of smart technology ensures green growth. This finding is also backed by Kouton (2019), who denotes that smart technologies facilitate an online transaction that in turn promotes green growth. This means that ICT helps in providing automated and intelligent solutions in various segments such as manufacturing, agriculture, and power generations that pave paths toward sustainable green growth. Also, education helps in promoting green growth, but our findings show that education in not matter in promoting green growth.

**TABLE 3:** ARDL estimates of green growth and CO_2_ emissions.

	Green growth				CO_2_ emissions			
	Coefficient	Std. error	t-stat	Prob.	Coefficient	Std. error	t-stat	Prob.
**Short-run**								
ICTS	−0.015	0.005	2.843	0.010	−0.074	0.159	0.468	0.648
ICTS(-1)	0.008	0.005	1.530	0.142	−0.335	0.295	1.135	0.279
ICTS(-2)					0.383**	0.188	2.033	0.065
EDUCATION	−0.296	0.557	0.532	0.603	0.090**	0.041	2.218	0.047
EDUCATION(-1)					0.085*	0.046	1.852	0.089
EDUCATION(-2)					0.210***	0.049	4.292	0.001
REC	0.009	0.134	0.069	0.946	−0.014***	0.005	3.047	0.010
REC(-1)	0.441**	0.178	2.485	0.026	0.011*	0.007	1.673	0.120
FD	0.615***	0.105	5.816	0.000	−0.525	0.352	1.492	0.162
FD(-1)	−0.134	0.306	0.437	0.666	−0.429	0.278	1.540	0.149
TRADE	0.118**	0.051	2.306	0.037	0.007***	0.002	4.180	0.001
TRADE(-1)	0.001	0.065	0.005	0.996	0.002	0.002	1.265	0.230
TRADE(-2)	0.117**	0.055	2.132	0.051				
**Long-run**								
ICTS	1.284***	0.349	3.677	0.003	−0.020**	0.009	2.108	0.057
EDUCATION	0.279	0.534	0.522	0.610	−0.285***	0.014	20.90	0.000
REC	0.407**	0.179	2.270	0.040	−0.002	0.004	0.614	0.551
FD	4.845	9.406	0.515	0.615	−0.706**	0.307	2.295	0.041
TRADE	0.221***	0.040	5.515	0.000	0.007***	0.001	4.708	0.001
C	1.102	5.154	0.214	0.834	12.50	0.158	78.90	0.000
**Diagnostics**								
F-test	4.235*				7.145***			
ECM(-1)	−0.646***	0.138	4.692	0.000	−0.517***	0.102	5.049	0.000
LM	1.235				1.412			
BP	0.356				0.542			
RESET	1.012				0.562			
CUSUM	S				S			
CUSUM-sq	S				S			

***p < 0.01, **p < 0.05, *p < 0.1, respectively.

An increase in renewable energy consumption reports a positive increase in green growth with a coefficient estimate 0.407 percent. However, financial development brings no significant impact on green growth in China in the long-run. Green growth increases significantly due to an increase in trade. It implies that in response of a 1 percent upsurge in trade, green growth increases by 0.221 percent in the long-run. The findings recommend that such policies should be adopted that promote trade and renewable energy consumption, thus, results in flourishing green growth in the long-run. The green growth model’s short-run results show that ICT, education, and renewable energy consumption have insignificant effects. However, financial development and trade variables bring a positive and significant increase in green growth in the short-run.

The long-run results of the CO_2_ emissions model demonstrate that ICT and education contribute effectively in reducing CO_2_ emissions as shown by negative and significant coefficient estimates of both variables. It infers that a 1 percent increase in ICT reduces CO_2_ emissions by 0.020 percent, while a 1 percent upgrade of education reduces CO_2_ emissions by 0.285 percent in the long-run. Our findings are supported by Haini (2021); Li and Ullah (2021), and Usman et al. (2021). They confirm that ICT and education both can be used as effective policy tools for improving environmental sustainability. Our result is also backed by the Porter hypothesis, who infers that smart technology significantly reduces CO_2_ emissions. Our finding is also verdict by ecological modernization theory (Buttel, 2000), which reveals that ICT brings social-environmental transformation and positively changes the behavior of organizations and individuals regarding the environment. This means that ICT enhances efficiency and productivity of the production process resulting in CO_2_ emissions alleviation. While an advanced level of education facilitates eco-friendly innovation and promotes green technologies that control CO_2_ emissions. Our finding is also in line with Yao et al. (2019) found that higher education increases consumption of clean energy that causes a reduction in CO_2_ emissions. This means that highly educated and skilled labor force prefers to adopt clean energy production that protects environmental quality. Such as, Broadstock et al. (2016) denoted that highly educated households most likely prefer to use such appliances that consume relatively less energy and are more energy-efficient.

Renewable energy consumption reports an insignificant impact on CO_2_ emissions in this model. CO_2_ emission tends to decline significantly due to an upsurge in financial development. It is shown that a 1 percent increase in financial development causes a 0.706 percent decline in CO_2_ emissions in the long-run. In contrast, CO_2_ emission intensifies significantly due to an upsurge in trade activity. It is shown that a 1 percent increase in trade causes 0.007 percent expansion in CO_2_ emissions in the long-run. The short-run results of CO_2_ emissions model infer that ICT reports no significant impact on CO_2_ emissions, while education intensifies CO_2_ emissions significantly. However, CO_2_ emission reduces due to an increase in renewable energy consumption in the short-run. Trade activity tends to enhance CO_2_ emissions in the short-run. The lower panel of Table 3 provides the findings of some important diagnostic tests to validate the outcomes of both ARDL models. In both models, the findings of F-tests and ECM tests confirm the cointegration association in the long-run among variables. The coefficient estimates of LM tests and BP tests are statistically insignificant, which confirms that our models are free from heteroskedasticity and autocorrelation. The outcomes from the causal analysis are informed in Table 4. The results display no causality between ICTs and green growth. While unidirectional causality exists from education to green growth, ICTs to CO_2_ emissions, and education to CO_2_ emissions.

**TABLE 4:** Results of causality tests in China.

Null hypothesis	F-stat	Prob.	Decision	Null hypothesis	F-stat	Prob.	Decision
ICTS → GG	0.725	0.496	No	ICTS → CO_2_	3.399	0.052	Yes
GG → ICTS	0.449	0.644	No	CO_2_ → ICTS	1.687	0.208	No
EDUCATION → GG	3.120	0.064	Yes	EDUCATION → CO_2_	4.572	0.022	Yes
GG → EDUCATION	1.615	0.222	No	CO_2_ → EDUCATION	0.286	0.754	No
REC → GG	0.940	0.406	No	REC → CO_2_	0.845	0.443	No
GG → REC	0.023	0.978	No	CO_2_ → REC	4.141	0.030	Yes
FD → GG	0.422	0.661	No	FD → CO_2_	0.028	0.972	No
GG → FD	0.168	0.846	No	CO_2_ → FD	5.915	0.009	No
TRADE → GG	0.372	0.694	No	TRADE → CO_2_	0.866	0.434	No
GG → TRADE	3.562	0.046	No	CO_2_ → TRADE	2.262	0.128	No
EDUCATION → ICTS	0.124	0.884	No	EDUCATION → ICTS	0.124	0.884	No
ICTS → EDUCATION	4.993	0.016	No	ICTS → EDUCATION	4.993	0.016	Yes
REC → ICTS	0.135	0.875	No	REC → ICTS	0.135	0.875	No
ICTS → REC	2.781	0.084	No	ICTS → REC	2.781	0.084	No
FD → ICTS	0.401	0.674	No	FD → ICTS	0.401	0.674	No
ICTS → FD	9.975	0.001	No	ICTS → FD	9.975	0.001	No
TRADE → ICTS	0.311	0.736	No	TRADE → ICTS	0.311	0.736	No
ICTS → TRADE	0.160	0.853	No	ICTS →TRADE	0.160	0.853	No
REC →EDUCATION	0.006	0.994	No	REC → EDUCATION	0.006	0.994	No
EDUCATION → REC	6.789	0.005	Yes	EDUCATION → REC	6.789	0.005	Yes
FD → EDUCATION	0.738	0.490	No	FD → EDUCATION	0.738	0.490	No
EDUCATION → FD	4.816	0.018	No	EDUCATION → FD	4.816	0.018	No
TRADE → EDUCATION	1.779	0.192	No	TRADE → EDUCATION	1.779	0.192	No
EDUCATION → TRADE	0.588	0.564	No	EDUCATION → TRADE	0.588	0.564	No
FD → REC	2.390	0.115	No	FD → REC	2.390	0.115	No
REC → FD	0.961	0.398	No	REC → FD	0.961	0.398	No
TRADE → REC	1.406	0.266	No	TRADE → REC	1.406	0.266	No
REC →TRADE	0.840	0.445	No	REC → TRADE	0.840	0.445	No
TRADE → FD	0.831	0.449	No	TRADE → FD	0.831	0.449	No
FD → TRADE	1.041	0.370	No	FD → TRADE	1.041	0.370	No

## Conclusion

China has witnessed a fast escalation of ICT diffusion in terms of mobile phone subscriptions and internet users in recent years. The escalation in ICT diffusion poses job creation, economic and environmental development. A rapid increase in ICT diffusions crucially affects green growth in the economy. The role of human capital is continuously increasing in China in the field of production in this era of competition and globalization. An increasing level of education promotes the earnings of households consequently increasing green economic growth. Furthermore, skilled and educated households prefer to adopt low carbon-based appliances that lead to a reduction in CO_2_ emissions. Previous studies have not adequately explored the role of ICTs diffusion and human capital on green growth. For this purpose, our study intends to explore the impact of ICTs diffusion and human capital on environmental and green growth performance in China for the period 1990 to 2019 by applying the ARDL approach. Findings of the green growth model reveal that ICT improves green growth while education produces an insignificant impact on green growth in long-term. Findings of the CO_2_ model display that ICTs and education both factors bring significant reductions in CO_2_ emissions in the long-run. The findings show that renewable energy consumption and trade result in increasing green growth in the long-run. Financial development and trade result in reducing CO_2_ emissions in the long-run.

Based on empirical findings, firstly, there is a need to improve the efficiency of energy in ICTs sector which could help in achieving green growth. Secondly, renewable energy consumption share should be increased in total energy consumption which could help in reducing CO_2_ emissions. The government of China should impose restrictions on high energy consumption-based equipment and should encourage e-commerce in the trade of ICT products. Thirdly, the Chinese government should examine the technological innovation, production, and consumption that ICT conveys and also ensure that the technological innovation and research and development offset the production and consumption benefits to attain green growth and improvement in environmental quality. Fourthly, investment in human capital should be increased that promote green economic growth and protect the environment. It is suggested that government should invest in environmental efficiency and environmental technologies simultaneously with human capital that could significantly contribute to pollution reduction. Lastly, policies to increase human capital should be implemented simultaneously with policies to promote ICTs contribution in order to confirm green growth and environmental protection.

The limitation of the study is that its conclusion and policy implications apply at a country level and these analyses do not take into consideration the provinces of China. There is a difference in growth patterns at a provincial level in China. Thus, there is a need to explore the same analysis for provincial levels as well. The study explores the symmetric relationship among variables, in future studies, asymmetric relationships among variables can be explored by adopting the NARDL approach.

## Data availability statement

The original contributions presented in this study are included in the article/supplementary material, further inquiries can be directed to the corresponding author.

## Author contributions

SC: conceptualization, methodology, software, and writing—original draft. MS: supervision and final draft approval, data collection and analyzing, and editing. MY: visualization and investigation. All authors contributed to the article and approved the submitted version.
